# The Effect of Needle Tract Nursing Methods to Reduce Needle Tract Infection in Patients with Indwelling Percutaneous Bone Puncture

This article has been retracted.

**DOI:** 10.1155/2021/5812562

**Published:** 2021-09-30

**Authors:** Weichao Li, Qiongshan Liu

**Affiliations:** ^1^The Seventh Affiliated Hospital, Sun Yat-sen University, Guangzhou, China; ^2^Infectious Diseases Department, Sun Yat-sen University, Guangzhou, China; ^3^The Office of Organ Donation and Transplant, Sun Yat-sen University, Guangzhou, China

## Abstract

Percutaneous bone piercing needles are used in orthopedics, which play the role of needle fixation. Needle tract infection is a common complication during the use of percutaneous bone needles. How to prevent needle tract infection is an important topic, so it is necessary to explore better needle tract care methods during percutaneous bone needle indwelling, to provide a basis for clinical work. Based on this, the purpose of this article is to study the effects of needle tract nursing methods for patients with indwelling percutaneous bone puncture needle infections. In this article, through an overview of percutaneous bone needle tract infection, on this basis, a detailed analysis of its occurrence, causes, and main influencing factors are carried out. Experimental studies have shown that the incidence of needle tract infections is 23.64%, mainly mild needle tract infections. Mild needle tract infections account for 84.62% of all needle tract infections, of which grade 1 needle tract infections account for 50.00 of mild needle tract infections. Severe needle tract infections accounted for 15.38% of all needle tract infections. All severe needle tract infections were grade 4 needle tract infections. No patients had bone infections or osteomyelitis.

## 1. Introduction

Percutaneous orthopedic needles are metal rods or needles used for external fixation and bone dispersion devices. They have been used to treat fractures for a century and are still widely used in orthopedics [1, 2]. The percutaneous bone needle passes through the skin, close to the muscle and soft tissue, and finally enters the bone tissue, or stays in the bone tissue, and passes through the other end of the bone [3, 4]. Needle tract infection is a common complication when using percutaneous bone puncture needles. Due to the different criteria for identifying needle tract infections, the needle tract infection rates reported in the literature vary greatly [5, 6]. After external fixation, due to the destruction of the integrity of the skin, the natural barrier of infection, needle tract infection has become a common postoperative complication of external fixation, which will lead to loosening of fixation, osteomyelitis, and failure of fixation. It is reported that the incidence of needle tract infection is about 21%–42%. Infection usually first involves the soft tissue around the needle path, and when it spreads to the deep, it will involve the bone. There is no unified standard for clinical diagnosis of needle tract infection. At present, it is largely based on clinical experience, with low reliability, and there is a lack of consensus in early diagnosis.

Scholars at home and abroad have conducted some research on how to reduce the infection of percutaneous bone puncture needle tract and do a good job in needle tract care. The initial research focused on the choice of disinfectant. The current research on disinfectants focuses on two aspects, namely, the comparison between sterile disinfectants and cleaning agents (such as soapy water) and the comparison between various sterile disinfectants. While comparing the effects of various disinfectants, some scholars have conducted comparative studies on conventional and unconventional disinfection of needle tracts. Studies by Patterson et al. have shown that there is no significant difference in the infection rate of the needle tract between patients with conventional and unconventional disinfection of the needle tract; that is, there is insufficient evidence to prove that disinfecting the needle tract has an effect on the prevention of needle tract infection [7]. The correct diagnosis of soft tissue or bone tissue infection depends on tissue specimen culture, but it should be noted that the specimen culture results collected on gauze or emergency treatment of open fracture are meaningless for the diagnosis of infection. When the sensitivity and specificity of total leukocyte count and leukocyte classification for the diagnosis of needle tract infection are not high, molecular biological indicators have an important reference value.

In summary, percutaneous orthopedic needles are widely used in clinics, and needle tract infection is the main problem in their use. Although many studies have been conducted on the prevention of needle tract infections at home and abroad, the current literature does not have enough evidence to prove the most effective method of needle tract care, and there are no standardized regulations, clinical practice standards, or corresponding nursing care on how to reduce needle tract infections. Redness and swelling around the needle path is not the basis of needle path infection, but redness and swelling around the needle path combined with exudation is an important indication of needle path infection.

## 2. Application Research on Needle Tract Nursing Methods to Reduce Needle Tract Infection in Patients with Indwelling Percutaneous Bone Puncture Needles

### 2.1. Overview of Percutaneous Bone Needle Tract Infection

#### 2.1.1. What Happened

The most common bacteria that cause needle tract infections are *Staphylococcus aureus* and *Staphylococcus epidermidis*. In the process of indwelling percutaneous needle puncture, the needle tract may be contaminated with *Staphylococcus aureus* and cause needle tract infection. The emergence of *Pseudomonas aeruginosa* may be caused because most of the patients used antibacterial drugs after the operation, and most of the pathogens were controlled. She is a pathogen with strong drug resistance. Once the patient's resistance drops, it is easy to cause drug-resistant bacteria.

#### 2.1.2. Cause of Occurrence

The aseptic inflammation formed after percutaneous bone needle insertion develops into infectious inflammation, and the bacterial biofilm plays a vital role. Biofilm is a bacterial colony structure formed by the coating of extracellular polymer secreted by bacterial cells. It can help bacteria adhere to biological or nonbiological surfaces. Studies have shown that after the formation of biofilms, bacteria produce strong resistance under environmental pressures, such as nutritional deficiencies and decreased body resistance, so that pathogenic bacteria can survive. It is considered that pathogenic microorganisms cause disease in humans. An important risk factor, the process of biofilm formation is relatively complicated, and it is mainly divided into three stages:

1. Bacterial adhesion period: reversible floating state
2. Irreversible growth period: bacteria grow and multiply to form microcolonies that gradually thicken and accumulate
3. Maturity stage: the formation of a heterogeneous three-dimensional structure; finally the bacteria are released from the surface of the biofilm or carrier to spread and colonize new other surface materials

Whether needle tract inflammation develops from aseptic inflammation to infectious inflammation depends on the dynamic balance between the bacterial biofilm and the body's resistance. Therefore, the development process of needle tract infection is related to the three stages of biofilm formation. If the resistance of the human body declines, bacterial proliferation in the needle tract will occur first, and then it will develop into a needle tract infection. With the further decline of the body's resistance or excessive nutritional deficiency, not only mild needle tract infections but also severe needle tract infections and even infections of other parts of the body may occur.

Needle tract infection is very common. On average, there is one needle tract infection with an external fixator every month. Most needle tract infections are superficial skin infections, which can be easily cured by taking antibiotics. The early manifestation of needle tract infection is the aggravation of local pain. The pain worsened rapidly in the following 6 to 12 hours. Other needle characteristics, such as secretions, erythema, and skin changes, are easy to mislead parents.

### 2.2. Main Influencing Factors of Needle Tract Infection

#### 2.2.1. Stability of Percutaneous Bone Needle

Loosening of the needle track occurs as a result of a continuous increase in bone stress. Mahan et al. carried out statistics and analysis on 42 cases (214 percutaneous bone piercing needles) of external fixation treatment of tibia, radius, and femur patients. The results showed that 75% of patients had bacterial proliferation, 71% of patients had needle tract cultured nonpathogenic bacteria, and of patients with loose needle tract, 82% of patients had needle tract cultured pathogenic bacteria. The conclusion is that the loose needle track can predict the existence of pathogenic bacteria, and the loose needle track is the most important risk factor for needle track infection [8]. Ning Rongxiang and others counted 50 cases of tibia and fibula fractures treated with external fixation from February 2002 to February 2006. The incidence of needle tract infection was 15%, and the incidence of needle tract loosening was 10% [9]. Oral antibiotic treatment is started when there are early signs of needle tract infection. The main antibiotics include cephalexin and cotrimoxazole; adjuvant antibiotics include cotrimoxazole and clindamycin; and the third antibiotic includes ciprofloxacin.

#### 2.2.2. Indwelling Site of Percutaneous Bone Needle

Many scholars at home and abroad have proposed that needle tract infection is related to the location of percutaneous bone needle indwelling. The Sims study reported the needle tract infection rate of different parts of the percutaneous bone needle. The femoral needle tract infection rate was 87%, the needle tract infection rate around the knee joint was 82%, and the tibia needle tract infection rate was 70%. The results show that the needle tract infection rate is higher near the heart, near the joints, rich in soft tissue, or swollen [10]. Henry's study also showed the same result; that is, the infection rate of the needle tract in the femur is 35% higher than that in the tibia. It is also the percutaneous bone needle placed in the femur and the needle tract infection at the proximal end. The rate is higher than the middle and lower parts of the femur. In summary, the risk of percutaneous bone needle tract infection is higher in the proximal end, proximal joint, near open fracture wound, and soft tissue rich or swollen sites [11]. Swab culture can be carried out for needle tract infection resistant to conventional oral antibiotics: the culture results must use skin routine flora to correctly judge and analyze. The culture results are helpful to identify unusual flora, such as *Pseudomonas* and methicillin-resistant *Staphylococcus aureus*. The culture results are conducive to the selection of specific antibiotics for treatment.

#### 2.2.3. The Patient's Injury

Li Kanghua and others counted and analyzed 120 patients with severe open fractures treated with external fixation from 2000 to 2003. A total of 11 cases of needle tract infection occurred, and the needle tract infection rate was 9.2%. The more severe the patient's condition and the more complicated the complications, the higher the needle tract infection rate [12–14].

#### 2.2.4. Indwelling Time of Percutaneous Bone Needle

Studies have shown that the longer the percutaneous bone needle indwelling time, the higher the incidence of needle tract infection. Li Kanghua and others counted and analyzed 120 patients with severe open fractures treated with external fixation from 2000 to 2003. The results of the study showed that the difference between the latter two groups and the first group was statistically significant, that is, longer retention time.

### 2.3. Clinical Manifestations of Patients with Percutaneous Bone Needle

Severe needle tract infection is rare and usually occurs in the deep. (1) Severe infection begins with the pain of a typical needle tract infection and ends with progressive erythema. (2) General symptoms include fever, drowsiness, discomfort, and nausea. (3) It must not be ignored and must be treated immediately. (4) The patient was admitted to the hospital for intravenous antibiotics. (5) If the site of needle tract infection does not respond to intravenous antibiotics within 24 hours, it is necessary to enter the operating room, remove the needle and debridement, and curette the surrounding area. This article selects patients who were hospitalized in the orthopedic ward of a tertiary A hospital in a certain area who underwent percutaneous bone puncture treatment. Among them, the patients who were hospitalized from January to December 2019 were the control group (100 cases), and the patients who were hospitalized from January to December 2020 were the experimental group (120 cases). The types of patients' diseases are shown in Table 1 (*X*^2^/*t*: variance; *P* : statistical standards).

In addition, variance is a measure of the degree of dispersion when probability theory and statistical variance measure random variables or a group of data. In probability theory, variance is used to measure the deviation between random variables and their mathematical expectations (i.e., mean). Variance in statistics (sample variance) is the average of the square value of the difference between each sample value and the average of all sample values. In many practical problems, it is of great significance to study the variance, that is, the degree of deviation.

It can be seen from Figure 1 that the main disease types of the research subjects are 152 fractures, of which 70 are comminuted fractures and 60 are multisegment fractures. The type of injury is mainly closed injury, and the device used is mainly bone traction in 116 cases.

Based on the clinical analysis of disease types, the retention time of the patient's percutaneous bone puncture needles was tested by normal distribution shown as follows:

(1) $$\begin{array}{c} X∼N\left(\mu ,\sigma^{2}\right),\\ Y=\frac{X-\mu }{\sigma }∼N\left(0,1\right). \end{array}$$

The specific situation is shown in Table 2.

It can be seen from Figure 2 that the retention time of percutaneous bone piercing is normally distributed after inspection: the shortest time is 4 days and the longest time is 84 days, mainly concentrated in 15–28 days (75 cases, 34.09%) and 29–42 days (74 cases, 33.64%). The length of hospital stay of the patients showed a normal distribution after inspection. The shortest time was 14 days and the longest 84 days, mainly concentrated in 15–28 days (81 cases, 36.82%) and 29–42 days (84 cases, 38.18%).

### 2.4. Research Indicators and Measurement Methods

#### 2.4.1. General Patient Information

General information includes disease diagnosis, case number, injury type, device used, indwelling time, hospitalization time, percutaneous bone needle insertion time, removal time, admission date, discharge date, indwelling site and quantity, the time when the patient has needle tract infection, infection grade, and antibiotic usage.

#### 2.4.2. Evaluation Index of Needle Path Nursing Effect

*(1) The Incidence of Percutaneous Needle Tract Infection in Patients*. The patient's needle track and surrounding conditions were evaluated at 9 a.m. and 9 p.m. each day after the operation. On the 3^rd^ day, the 1^st^ weekend, the 2^nd^ weekend, the 4^th^ weekend, and the 6^th^ weekend after the operation, bacterial culture was performed on each needle path. In addition, whenever a patient is hospitalized, if there is any suspicion of infection in the patient's needle tract, a bacterial culture is done for the needle tract:
  (2) $$\begin{array}{c} \text{Incidence of needle tract infection}=\frac{\text{Amount of needle tract infection}}{\text{Total number of patients}}\times 100\%. \end{array}$$
*(2) Time of Percutaneous Needle Tract Infection in the Patient*. Record the time of the first needle tract infection after the operation, in days.
*(3) Needle Path Discomfort during Needle Path Care*. The evaluation time of the control group was at 9 a.m. and 9 p.m. each day after the operation. The evaluation time of the experimental group was evaluated whenever the nurse disinfected the needle path with saline and replaced the sterile gauze at the needle hole according to the patient's needle path and surrounding conditions. Needle path discomfort is expressed by the mean value ± standard deviation (*x* ± SD) of the discomfort during the evaluation period.
*(4) Bacterial Culture and Result Judgment*. Needle tract bacterial culture method: use a throat swab, smear around the needle tract opening, and then rotate the throat swab, try to touch the needle tract opening in all directions. If there is a secretion at the mouth of the needle, focus on retaining the secretion for culture. The sampling process follows the principle of aseptic operation to avoid contamination due to improper operation.

## 3. An Experimental Study on Reducing Needle Tract Infection in Patients with Indwelling Percutaneous Bone Puncture Needles

### 3.1. Research Objects

(1) Research population
  1. Overall study: patients treated with percutaneous bone puncture needles.
  2. Research sample: patients who were hospitalized with percutaneous bone needles in the orthopedic ward of a hospital from January 1, 2019, to December 31, 2020.
(2) *Sample Size Calculation*. Compare the required sample size according to the two sample rates; that is, the needle path uses 70% alcohol disinfection group (17.5%) once a day. Through the look-up table method, the total samples were 192 cases.

### 3.2. Research Methods

1. *Sampling Survey Method*. This experiment selected patients who were hospitalized in the orthopedics department of a tertiary A hospital in a certain area that met the conditions of this article, making the research results of this article more real and reliable. It is to select the survey units completely at random without any grouping, classification, queuing, and so on. The characteristics are the probability of each sample unit being selected is equal, each unit of the sample is completely independent, and there is no certain correlation and exclusion between them. Simple random sampling is the basis of other sampling forms. It can include isometric sampling, type sampling, and cluster sampling.
2. *Comparative Analysis Method*. In this experiment, the control group and the experimental group were set up for comparative analysis, and the results obtained were analyzed and researched using the analytic hierarchy process. These data not only provided theoretical support for the topic selection of this article but also provided data for the final research results of this article. The comparison method, also known as a comparative analysis method or comparative analysis method, is an analysis method to prompt the difference between the actual number and the base through the comparison between the actual number and the base, to understand the achievements and problems of economic activities. Comparative analysis is often used in scientific inquiry activities, which is similar to the equivalent substitution method.
3. *Mathematical Statistics*. Use relevant software to make statistics and analysis on the research results of this article.

## 4. An Experimental Analysis of Needle Tract Nursing to Reduce Needle Tract Infection in Patients with Indwelling Percutaneous Bone Puncture

### 4.1. Incidence and Severity of Needle Tract Infection

In order to make this experiment more scientific and effective, this experiment investigated and analyzed the incidence and severity of needle tract infections. The data obtained are shown in Table 3.

It can be seen from Figure 3 that the incidence of needle tract infections was 23.64%, with mild needle tract infections being the main ones. Mild needle tract infections accounted for 84.62% of all needle tract infections, and grade 1 needle tract infections accounted for mild needle tract infections 50.00%. Severe needle tract infections accounted for 15.38% of all needle tract infections. All severe needle tract infections were grade 4 needle tract infections. No patients had bone infections or osteomyelitis.

### 4.2. Analysis of the Time of Needle Tract Infection

In 52 patients with needle tract infection, the shortest time for needle tract infection occurred was the 4^th^ day after the operation, and the longest was the 42^nd^ day after the operation. For further analysis of the time when the needle tract infection occurred in 52 patients with needle tract infection; see Table 4.

Figure 4 shows that postoperative needle tract infections have two high-incidence periods. The first high-incidence period is the second weekend after surgery. There are 15 cases, accounting for 28.85% of the total number of needle tract infections. Two weeks after the operation, a scab gradually formed around the needle hole, which played a certain role in preventing needle tract infection, and then there was a downward trend in needle tract infection. The second-high incidence was the 6^th^ weekend after surgery, with 12 cases, accounting for 23.08% of the total number of needle tract infections. It is related to the increase of functional exercise and loose needle track.

## 5. Conclusion

Because the needle track injury rate in the control group is not only higher than that in the experimental group, it also increases the needle track discomfort during the needle track care process. Therefore, it is recommended that 75% of the sterile gauze is not routinely applied twice a day at 9 a.m. and 9 p.m. For medical staff, objective research results can be used to guide clinical work, promote medical-care cooperation, reduce nurse-patient conflicts, reduce unnecessary workload, and improve the quality of medical care. For patients, it can reduce needle tract discomfort, reduce the incidence of needle tract infection during needle tract care, and promote patient recovery. With the rapid development of big data, like computers and the Internet, big data is likely to be a new round of technological revolution. Emerging technologies such as data mining, machine learning, and artificial intelligence may change many algorithms and basic theories in the data world and achieve breakthroughs in science and technology.

## Figures and Tables

**Figure 1:** Type of disease.

**Figure 2:** Retention time.

**Figure 3:** Incidence and severity of needle tract infection.

**Figure 4:** Analysis of the time of needle tract infection.

**Table 1:** Type of disease.

	Research object	Control group	Test group	*X* ^2^/*t*	*P*
Limb lengthening	30	12	18	0.438	0.803
Fracture	152	70	82	—	—
Comminuted fracture	70	32	38	0.015	0.992
Multiple fracture	60	28	32	—	—
Ordinary fracture	22	10	12	—	—
Joint related diseases	38	18	20	—	—

**Table 2:** Retention time.

	Research object	Control group	Test group	*X* ^2^/*t*	*P*
0–7	14	8	6	6.809	0.146
8–14	36	22	14	—	—
15–28	75	30	45	—	—
29–42	74	29	45	—	—
42	21	11	10	—	—

**Table 3:** Incidence and severity of needle tract infection.

	Number of occurrences (*N*)	Incidence (%)
Level 1	22	10.00
Level 2	17	7.73
Level 3	5	2.27
Level 4	8	3.64

**Table 4:** Analysis of the time of needle tract infection.

	0–5	5–10	10–15	15–20	20–25	25–30	30–35	35–40	40–45
Man	1	1	8	2	1	4	2	2	5
Woman	0	1	7	3	2	3	1	1	7

## Data Availability

The data underlying the results presented in the study are available within the manuscript.
